The article "Detection of Dental Diseases through X-Ray Images Using Neural Search Architecture Network" was published in 2022. Journal: Comput Intell Neurosci.

# Detection of Dental Diseases through X-Ray Images Using Neural Search Architecture Network

**DOI:** 10.1155/2022/3500552

**Published:** 2022-04-30

**Authors:** Abdullah S. AL-Malaise AL-Ghamdi, Mahmoud Ragab, Saad Abdulla AlGhamdi, Amer H. Asseri, Romany F. Mansour, Deepika Koundal

**Affiliations:** ^1^Information Systems Department, Faculty of Computing and Information Technology, King Abdulaziz University, Jeddah 21589, Saudi Arabia; ^2^Information Systems Department, HECI School, Dar Alhekma University, Jeddah, Saudi Arabia; ^3^Information Technology Department, Faculty of Computing and Information Technology, King Abdulaziz University, Jeddah 21589, Saudi Arabia; ^4^Centre for Artificial Intelligence in Precision Medicines, King Abdulaziz University, Jeddah 21589, Saudi Arabia; ^5^Mathematics Department, Faculty of Science, Al-Azhar University, Naser City 11884, Cairo, Egypt; ^6^Medical Doctor, King Abdulaziz General Hospital, Jeddah, Saudi Arabia; ^7^Biochemistry Department, Faculty of Science, King Abdulaziz University, Jeddah 21589, Saudi Arabia; ^8^Department of Mathematics, Faculty of Science, New Valley University, El-Kharga, 72511, Egypt; ^9^School of Computer Science, University of Petroleum & Energy Studies, Dehradun, India

## Abstract

An important aspect of the diagnosis procedure in daily clinical practice is the analysis of dental radiographs. This is because the dentist must interpret different types of problems related to teeth, including the tooth numbers and related diseases during the diagnostic process. For panoramic radiographs, this paper proposes a convolutional neural network (CNN) that can do multitask classification by classifying the X-ray images into three classes: cavity, filling, and implant. In this paper, convolutional neural networks are taken in the form of a NASNet model consisting of different numbers of max-pooling layers, dropout layers, and activation functions. Initially, the data will be augmented and preprocessed, and then, the construction of a multioutput model will be done. Finally, the model will compile and train the model; the evaluation parameters used for the analysis of the model are loss and the accuracy curves. The model has achieved an accuracy of greater than 96% such that it has outperformed other existing algorithms.

## 1. Introduction

Tooth decay, sometimes referred to as dental caries, is a disease that affects millions of people in daily life [1]. Depending on the extent of the lesion, dental caries can be categorized as normal, initial, moderate, or extensive [2]. Early identification of dental caries can save money in the long run by avoiding more intrusive procedures. Bitewing radiography is the gold standard for diagnosing demineralized proximal caries, which is difficult to detect with clinical investigations alone [3]. Detecting proximal caries is made simple with bitewing radiography and a visual assessment. Fluorescence-based technologies like DIAGNOdent (KaVo Charlotte, NC, USA) and fiber optic transillumination can also be used to detect dental caries. The disadvantages of these approaches include their inability to detect posterior beginning proximal caries and the cost of additional devices. Therefore, bitewing radiographs are still the most often utilized approach in clinical settings [4].

Dental informatics is a new and rising topic in dentistry, which can improve treatment and diagnostics and reduce stress and tiredness during everyday practice. Dental procedures create a vast amount of data from sources like high-resolution medical imaging and biosensors with continuous output [5]. Dental professionals can benefit from using computer programs in various decision-making processes, including prevention, diagnosis, and treatment planning [6]. In clinical settings, deep learning is currently one of the artificial intelligence methods used [7]. Deep learning's success is mainly attributable to advances in computing power, enormous data, and new methods. This strategy has been proven in image-based diagnostics and is widely utilized [8]. During the last decade, deep learning-based applications have exploded in popularity. Convolutional neural networks (CNNs) have become a popular choice for medical image analysis because of their rapid development. Clinical skin screenings, mammography, and eye exams for diabetic retinopathy have successfully used CNNs. Hence, CNNs have been particularly successful in the field of a cancer diagnosis [9].

Dental caries can be difficult to diagnose with radiographs, even though they are widely accepted as a diagnostic tool [10]. Even when utilizing the same radiograph, observers have significant discrepancies regarding whether caries lesions are seen. The inter-rater agreement can be affected by factors such as the radiograph's quality, how the dentist views it, and the time it takes to complete each exam. The mean kappa values for the presence or absence of dental caries and their degree ranged from 0.30 to 0.72 when 34 raters examined the identical bitewing radiographs in a prior study. Consistency is a significant issue, especially when detecting the early stages of dental caries.

Researchers have recently extensively investigated the use of deep learning and convolutional neural networks (CNNs) to interpret various types of medical images, with promising results [11]. There has been a rise in deep learning in diagnosing diseases, which has resulted in improved clinical outcomes. Using deep convolutional networks in dentistry has been studied since 2015.

The organisation of the paper is as follows: Section 2 discusses the literature survey. In Section 3, the proposed methodology has explained, and Section 4 covers the results and discussion. In Section 5, the conclusion and future work are mentioned followed by the reference section.

## 2. Related Work

Computer-aided image segmentation in dentistry has been introduced in the literature using various techniques [12, 13]. Image classification and object detection are two examples of computer vision problems used by deep learning. A growing use of deep learning-based algorithms has recently been becoming popular for image segmentation. Full-connected networks (FCNs) are a common segmentation approach that can be used in various imaging applications.

By employing 1500 panoramic X-ray radiography, Jader et al. [14] developed the profile of each tool using a mask region-based convolutional neural network. Accuracy, F1-score, precision, recall, and specificity were used as outcome metrics in this investigation, with 0.98, 0.88, 0.94, 0.84, and 0.99, respectively. Muramatsu et al. [15] used a fourfold cross-validation method using 100 dental panoramic radiographs to build an object detection network. As a result, 96.4% and 93.2% were the sensitivity and the accuracy of tooth detection, respectively. Miki et al. [16] used an AlexNet-based convolutional neural network (DCNN) to classify dental cone-beam computed tomography (CBCT) pictures of tooth kinds. Researchers used 42 images to train the network and ten images to test it and achieved an accuracy rate above 80% in that study. Furthermore, TensorFlow tool package has been employed by Chen et al. to identify and count teeth in dental periapical videos using quicker R-CNN features [17]. In this case, 800 images were used for training, 200 for testing, and 250 for validation. There was a correlation between the result metrics of recall and precision (0.728 and 0.771, respectively). They used a neural network to forecast the number of missing teeth.

Zhang et al. [18] used periapical images with Faster RCNN and R-FCN (region-based fully convolutional networks). A total of 700 images were used to train the network, 200 for testing, and 100 for validation. The model has produced a precision of 95.78% and a recall of 0.961. Velemínská et al. [19] compared the accuracy of an RBFNN and a GAME neural network in estimating the age of the Czech population between the ages of three and seventeen. A panoramic X-ray of 1393 people ranging in age from three to 17 years was used in this investigation. To get an idea of the variance, the standard deviation was used. Afterwards, Tuzoff et al. [20] used a Faster R-CNN architecture and 1352 panoramic images to detect teeth [3]. A sensitivity of 0.9941 and a precision of 0.9945 were achieved in this study. Schwendicke et al. have implemented Resnet18 and Resnext50, and CNNs were trained and validated using a 10-fold cross-validation method. One-cycle learning rate policy was applied, with the minimum learning rate of 105 and maximum learning rate of 10-3, respectively, during the training process. PPV/NPV and AUC (area under the receiver operating characteristic curve) were some of the metrics used to evaluate the model's performance. To see if the CNNs were based on features that dentists would also use, feature visualisation was used. Approximately 41% of the teeth were found to have caries lesions. Raith et al. [21] identified teeth using a CNN architecture and the PyBrain package, achieving a performance of 0.93. Based on the tooth type (molar, incisor, or premolar), an AlexNet database of 100 panoramic radiographs was used by Oktay to recognize teeth with an accuracy of above 0.92 [22].

Fukuda [23] has used panoramic radiography and a convolutional neural network (CNN) technology, and this study attempted to determine whether or not VRF could be detected. In this method, 330 VRF teeth with clearly visible fracture lines were picked from the hospital imaging database in 330 panoramic images. Two radiologists and an endodontist confirmed the presence of VRF lines. Of the 300 images, 240 images were assigned to a training set and 60 images to a test set, respectively. CNN-based deep learning models were created using DIGITS version 5.01 to detect VRFs. The implemented method has achieved a precision of 0.93, and the F measure was 0.83. Though a number of works have been presented on the detection of the object of interest from the dental X-ray images, still there is a need for an automated technique that can detect the desired objects accurately and effectively.

It was demonstrated that SegNet [24] could be trained more quickly using an encoder-decoder architecture. Encoder-decoder architecture with skip links between upsampling and downsampling layers allowed the U-Net network to combine high-resolution characteristics with an encoded and decoded output. Some U-Net versions, such as 3D U-Net [25], V-Net [26], and attention U-Net [27], have also been proposed to improve performance. According to Fan et al. [28], an efficient network called PraNet was developed to balance inference speed with segmentation accuracy. In addition to the above-mentioned general frameworks for picture segmentation, multiple deep learning-based algorithms have been used to segment X-ray pictures. Al-Antari et al. directly segmented live using the DeepLab [29]. To detect COVID-19 infections from chest X-ray images, Blain et al. presented a modified UNet network [30]. Moeskops et al. trained a multitask segmentation model using a variety of visual modalities [31]. RNN was first integrated into FCN by Trullo et al. as a conditional random field module [32–34].

## 3. Materials and Methods

### 3.1. Datasets

The dental image dataset consisted of unidentified and anonymized panoramic dental X-ray images of a total of 116 patients, acquired from Noor Medical Imaging Center, Qom, Iran. This dataset covered different dental conditions of teeth from healthy to partial and complete edentulous cases. All conditions of different cases are segmented by two dentists manually. The dataset can be obtained from the Kaggle website which is publicly available at https://www.kaggle.com/daverattan/dental-xrary-tfrecords.

### 3.2. Proposed Methodology

In this work, X-ray images of teeth will be used for performing the multiclass classification. In this classification, there are three classes such as “cavity,” “filling,” and “implant.” In the initial phase, the proposed work will augment the data and then preprocess it. Next, the data are split into training and validation sets. Finally, the multioutput model is developed which is used to compile and train the model.  Figure 1 illustrates the flowchart of the proposed work.

#### 3.2.1. Data Augmentation

The data augmentation has been done by applying different types of operations such as scale, rotates, translate, Gaussian blur, and Gaussian noise. The function has been defined to apply the augmentation such as bounding_box and image_aug. Therefore, before performing the augmentation, the dataset was of size 83, and after the augmentation, it has been increased to 245. The augmentation of the dataset has been done to increase the size of the dataset, so that more accurate results can be obtained.

#### 3.2.2. Preprocessing of the Image Dataset

The dataset is preprocessed by scaling the boundary box in the range of 0 to 1 so that model can understand easily. Some more resizing operation is also performed such as label_encoder, integer_labels, and onehot_labels. label_encoder is used to convert the textual data into numerical form, so that model can understand it in a better way. onehot_labels are used to convert the categorical data into numerical data.  Figure 2 illustrates the images of different types of teeth diseases.

Splitting the dataset: the dataset is split into the training set and the validation set. 90% of the data are taken as the training dataset, and 10% of the data are used for the validation purpose.

#### 3.2.3. Construction of the Multioutput Model

In this work, the transfer layer has been implemented by using a convolutional neural network. The convolution neural network has been constructed by incorporating different number of max-pooling layer, dropout layer, and activation functions.  Figure 3 shows the architecture of the proposed model in which the image matrix has been passed through the convolution feature map. The pooled representation of the features has been inserted in the fully connected dense layer, and then, finally, the activation function has been applied to perform the multiclass classification.

#### 3.2.4. Proposed NASNet Model

It is a machine learning model known as Neural Search Architecture Network (NASNet). Because it departs from established models like GoogleNet in several crucial ways, it has the potential to be a game-changer for artificial intelligence. In the context of neural network development, we expect it to perform at its highest level. To develop the most efficient architecture, one needs to have extensive knowledge of the subject matter.

Constructing neural networks requires a lot of trial and error, which may be very time-consuming and costly. Human professionals may have built a successful model architecture, but this does not guarantee that we have explored the whole network architectural space and found the optimal solution. Automated network architecture design has been made possible by the neural architecture search (NAS). It is a search algorithm that seeks the best method to accomplish a specific task. Many new proposals for faster, more accurate, and less expensive neural architecture search (NAS) approaches have sprung up in response to the ground-breaking work done in 2017 by Zoph & Le and Baker et al. [24]. For example, Google's AutoML and Auto-Keras are commercial services and open-source tools that make NAS accessible to the broader machine learning community. There are three important steps in the NASNet, which are search space, searching method, and estimation methodology.

Figure 4 represents the NASNet model in which there are two different cells; one is a normal cell, and the other one is a reduction cell. These cells are passed through different types of max-pooling layers, dropout layers, dilated convolutions, depth-wise separated convolutions, and the activation function. By using fewer floating-point operations and parameters than comparable architectures, the NASNet achieves state-of-the-art performance.

## 4. Results and Discussion

The discussed work is implemented using the Python programming language. The performance parameters used for the validation of the models are accuracy and loss. The proposed Model has achieved an accuracy of 96.51% with data augmentation and 93.36 without augmentation.  Table 1 lists the comparison of the proposed NASNet model with AlexNet and convolutional neural network. From Table 1, it has been observed that the NASNet model outperformed the AlexNet by 4.36% and CNN by 1.36% without any augmentation. It has also been observed from results that accuracy of 96.51% has been achieved by the proposed NASNet model by outperforming the AlexNet having 93% accuracy and CNN having 95% with data augmentation.  Figure 5 displays the comparison graph of the proposed model with the existing models.

Figure 6 shows the graph based on output accuracy and the output loss. The 10000-epoch iteration has been done to compute the accuracy and the loss of the proposed model. The proposed model has computed the loss of 0.0407.  Figure 7 illustrates the predicted image with implant class.

## 5. Conclusion

This paper proposes a method to perform multiclass classification through X-ray images. The work has implemented the convolutional neural network with a transfer learning approach, that is, NASNet. There are three different types of classes: cavity, filling, and implant used during the classification process. These assessments show that the procedure can be an initial stage in clinical practice processing and analysing dental pictures. The limited training dataset of 116 patient images is also a factor in the success of this approach. Image processing stages are applied to the neural networks with multiple max-pooling layers, dropout layers, and activation functions. While the goal of this work is to segment tooth instances, the strategy given here can be applied to similar challenges in other domains, such as separating cell instances. In the future work, the multiclass classification can be done in large datasets with a greater number of classes. A new advanced deep learning based on hybrid deep learning can be implemented that can enhance the existing performance.

## Figures and Tables

**Figure 1:** Flowchart of the proposed work.

**Figure 2:** Different types of images based on teeth disease.

**Figure 3:** Architecture of the proposed model.

**Figure 4:** NASNet model.

**Figure 5:** Comparison graph of the implemented model.

**Figure 6:** Graph of output accuracy and output loss.

**Figure 7:** Teeth image predicted with the implant class.

**Table 1:** Comparison of the proposed model with the existing model.

Models	AlexNet (%)	Convolutional neural network (%)	NASNet model (%)
Accuracy without data augmentation	89	92	93.36
Accuracy with data augmentation [33]	93	95	96.51

## Data Availability

Data are publicly available in Kaggle (https://www.kaggle.com/daverattan/dental-xrary-tfrecords).
